# A Data Mining Algorithm for Association Rules with Chronic Disease Constraints

**DOI:** 10.1155/2022/8526256

**Published:** 2022-08-23

**Authors:** YanRong Liu, LiJun Wang, Rong Miao, HengNi Ren

**Affiliations:** College of Information Engineering, Shaanxi Institute of International Trade & Commerce, Xi'an 712046, China

## Abstract

The Apriori algorithm in association rules is the main algorithm used in the treatment and prevention of chronic diseases in data mining, and the algorithm in the current stage of China's medical field of association between chronic diseases has some problems, such as the need to scan the transaction database of cases several times, producing a large data set and more redundant rules. To address the above problems, a data mining algorithm of association rules combining clustering matrix and pruning strategy is proposed, which improves the algorithm by using the clustering matrix method to compress the stored transaction database and introducing the prepruning and postpruning strategy methods on the basis of adding constraint conditions. The experimental results show that the optimization algorithm has unique advantages in reducing the number of database scans and the number of candidate item sets generated and ultimately greatly reduces the running time and I/O load of the algorithm, and the running efficiency of the algorithm is greatly improved.

## 1. Introduction

With the development of digital technology today, behind it is the support of powerful computer technology. Powerful computer technology must rely on massive databases. Computer database application technology has penetrated many aspects of people's lives, such as online shopping, smart home appliances, pathological analysis, prevention, etc. Extensive application is bound to produce a large amount of data. How to quickly find potentially useful information in this massive data has been a major problem that people are facing. Data mining technology can help people discover the knowledge hidden behind massive data. Driven by various medical and health modes, data mining technology has shown good application value and attracted more and more experts and scholars' attention. The improvement of information technology has also brought about the wide application of various medical systems. In the medical field, big data has also begun to be applied, and the data collected in various medical systems are of great research value for medical research and the diagnosis and treatment of chronic diseases. However, at present, all hospitals only collect and store patients' medical data without in-depth analysis and effective use, let alone using these data to analyze and mine the knowledge behind them. Using data mining technology to discover the hidden relationship from these medical data and provide services for doctors' clinical diagnoses has become a problem that researchers pay much more attention to.

In medicine, there is a lot of unknown information hidden behind the sign data [1] of patients with chronic diseases, which can provide a correct prediction for early diagnosis through data mining. Therefore, data mining technology has become an indispensable part of the hospital evaluation system and medical research. Methods of data mining techniques such as association Rules Mining, rough set theory [2], machine learning, and neural network [3] have their own advantages and disadvantages in medical data mining [4]. Among the many application fields of data mining, a promising research direction is the data mining algorithm of association rules which has been widely applied to e-commerce, prevention of chronic diseases [5], telecommunications industry, and insurance industry. Whether the association rule algorithm is good or bad in practice is shown by the final result of any system. Therefore, the study of the association rule algorithm is to study whether the association rules generated by it have greater relevance and whether they can help human intelligent life.

In the medical data analysis of chronic diseases, many scholars have applied the data mining technology of association rules to it and have achieved remarkable experimental results. Xu and Xu [6] used the characteristics of a numerical attribute of aggregation algorithm to discrete the data set and divided it into several optimized data sets, mining useful association rules in tumor diagnosis data and providing important reference value for clinical diagnosis of chronic cancer. Serbanati [7] established a prediction model for chronic disease patients using labor neural network and Logistic regression analysis technology, which provided a good prediction effect for chronic diseases such as hypertension and diabetes. Zhang et al. [8] used the classification algorithm to analyze the data of type I diabetes patients and found that the generated classification association rules were highly consistent with the results of medical research. The classification association rule technique has a good theoretical basis in the study of chronic diabetes. Zhou et al. [9] summarized the traditional Apriori algorithm and found that its biggest defect was that frequent item sets could be obtained only after repeated scanning of the database, which would inevitably affect the efficiency of data mining and occupy a large amount of memory. Wen et al. [10] put forward a kind of an association rule data mining algorithm combining matrix and index sort is proposed, the algorithm can delete useless transaction data and item sets in a transaction database, then the set of a frequent binomial is obtained by the product of matrix. Finally, the frequent item sets are obtained, the algorithm can directly find the frequent item sets are the biggest advantage of scanning the database. Although the efficiency of data mining has been improved, the database needs to be updated continuously during the mining process, which increases the time overhead of I/O. To sum up, although the theoretical research on the mining technology of association rules has been applied in many aspects, there is still a problem that effective association rules can not be quickly obtained during mining, which will have a great impact on the accuracy of the system association. Therefore, the research data mining algorithm of association rules is of great significance to people's convenient life.

## 2. Association Rule

### 2.1. Knowledge about Association Rules

The relevant definitions are as follows.

**Definition 1 .**

Suppose there is a set of items as follows: *A*={*a*_1_, *a*_2_, *a*_3_,…, *a*_*n*_}, *D* is the transaction database collection. Both *M* and *N* are nonempty subsets and both belong to *A*, and *M*⟶*N* is an expression in the form of an association rule. In the expression, *M* ⊂ *A*, *N* ⊂ *A*, and the intersection of *M* and *N* is not equal to the empty set. If *M* contains *k* number of sets, it is called *k*-item sets.

**Definition 2 .**

Suppose (*M*⟶*N*) is the ratio of the number of tuples containing *M* to the number of tuples containing *N*, and the result is expressed as a percentage [11], as shown in the following formula:

(1) $$\begin{array}{c} S\left(M⟶N\right)=\frac{\text{count}\left(M\cap N\right)}{\text{count}\left(D\right)}\times 100\%. \end{array}$$

**Definition 3 .**

(confident). refers to the percentage that the database contains transactions N even if it contains one transaction *M* , namely, the trustworthiness of the value [11]. The definition pattern of (confident) (*M*⟶*N*) is (confident) (*M*⟶*N*) represents the percentage of tuples containing *M* and *N* in tuple *M*, as shown in the following formula:

(2) $$\begin{array}{c} C\left(M⟶N\right)=\frac{S\left(M\cap N\right)}{S\left(N\right)}\times 100\%. \end{array}$$

**Definition 4 .**

Let min_supp be the minimum support threshold [12] and min_conf the minimum confidence threshold [13]. Assuming that there is an association rule in *D* that satisfies formulas (3) and (4), it is a strong association rule in *D* [14, 15]. The set that satisfies formula (3) is called frequent item sets, and the set that does not satisfy formula (3) is called infrequent item sets [16].

(3) $$\begin{array}{c} S\left(M⟶N\right)\geq \min\_\text{supp,} \end{array}$$

(4) $$\begin{array}{c} C\left(M⟶N\right)\geq \min\_\text{conf.} \end{array}$$

### 2.2. Apriori Algorithm

Apriori algorithm is one of the most widely used algorithms in association rule data mining. Such as medical system, commercial system, and the association rules generated by this algorithm are single-level, Boolean type [17] association rules in terms of classification. Apriori association rules algorithm scans the transaction database by a layer-by-layer iterative method and then obtains frequent item sets. The main idea of generating frequent item sets is as follows [18, 19]: first, scan the transaction database multiple times to generate candidate item sets of length *k*+1 from *k* frequent item sets; then, perform mining and judgment on *k*+1 candidate item sets to obtain *k*+1 Frequent item sets. According to the same method, until no more *k*-item sets are found, the algorithm execution ends.  Table 1 is the definition symbols in the algorithm.

The first stage of Apriori algorithm execution is to scan the transaction database to find out the support of each element in the candidate item sets *C*_*k*_ to determine whether the element joins *L*_*k*_ or not. If the generated frequent item set is a large item set containing 12 items, the minimum number of times to scan the transaction database is 12. When the larger the transaction database is, the larger the I/O load is; in the second stage of algorithm execution, the frequent item sets *L*_*k*−1_ generating the candidate item sets *C*_*k*_ is exponentially growing, and if the length of the frequent pattern is 200, the minimum number of postoption item set is 2^100^.When the candidate 2-item sets are larger, the final result is very considerable. When there is a large amount of data in the transaction database, the min_supp threshold and the min_conf threshold are set too small, and a large number of redundant rules will be generated [20], and with the increase of data in the transaction database, the generated association rules and he numbers grow exponentially. In order to improve the execution efficiency of the algorithm, this paper proposes an algorithm that combines a clustering matrix and pruning strategy under the condition of setting project constraints. The algorithm is optimized on the basis of the traditional Apriori algorithm, which will greatly improve the execution efficiency of the algorithm.

## 3. A Data Mining Algorithm with Item Constraints

The knowledge discovery of traditional association rule algorithm is achieved by setting min_supp and min_conf. A single setting of min_supp and min_conf results in more association rules, and a large part of them are redundant rules, and fewer rules meet the conditions. If the user can guide and control the mining process, the number of valid association rules can be increased, and the efficiency of mining can be ameliorated. Setting appropriate item constraints in the mining process can achieve better results and thus obtain effective association rules. In the research of this paper, first stage, preconstraints (hypertension, diabetes, etc.) are added to the database before generating frequent item sets to constrain the database; second stage, fundamentally reduce the frequency of database scans; the association rules that do not meet the set conditions are dropped. The above idea of applying preconstraints and postconstraints is applied to the generated Apriori algorithm, and Figure 1 shows the detailed execution flow of the algorithm.

### 3.1. The Main Idea of an Apriori Algorithm with Item Constraints

In the analysis of the previous section, the existing problems of the traditional Apriori have been clarified. The research in this paper is to add constraints on the basis of the traditional algorithm, use the cluster matrix compression storage method to store the transaction database, and obtain the candidate items by operating the matrix vector. Then, before the frequent item sets are self-connected, the pruning method is used to delete the item sets that do not meet the conditions. At this time, the redundant candidate item sets generated by the pruning strategy will be greatly reduced, thereby improving the data mining efficiency.

#### 3.1.1. Matrix Vector Strategy

The following definitions are made in the transaction database *D*.

**Definition 5 .**

The vector of *n*_*j*_ is denoted as *D*_*j*_, As shown in the following formula:

(5) $$\begin{array}{c} D_{j}=\left[\begin{array}{c} d_{1j}\\ d_{2j}\\ \vdots \\ d_{3j} \end{array}\right],\\ \text{where}d_{nj}=\left\{\begin{array}{c} 0,nj\notin D,\\ 1,nj\in D. \end{array}\right. \end{array}$$

The support frequency of *n*_*j*_ is as follows: support_*c*(*nj*)=∑_*n*=1_^*m*^*d*_*nj*_

**Definition 6 .**

The vector of the 2-term set {*i*_*i*_, *i*_*j*_} is denoted as *D*_*ij*_:

$D_{ij}=\left[\begin{array}{c} d_{1i}\wedge d_{1j}\\ d_{2i}\wedge d_{2j}\\ \vdots \\ d_{ni}\wedge d_{nj} \end{array}\right]$ , where, the symbol “ ∧” indicates the “AND” operation.

The support frequency of the 2-item set is as follows:

(6) $$\begin{array}{c} \text{support}\_c\left(\left\{i_{i},i_{j}\right\}\right)=\sum_{t=1}^{m}\left(d_{ti}\wedge d_{tj}\right). \end{array}$$

**Definition 7 .**

The vector of *k*_term set is denoted as *D*_1,2,…*k*_.

The support frequency of the *k*_term set is as follows:

(7) $$\begin{array}{c} \text{support}\_c\left(\left\{i_{1},i_{2},\ldots i_{k}\right\}\right)=\sum_{t=1}^{n}\left\{\left(d_{ti}\wedge d_{t2}\wedge \cdots \wedge d_{t\left(k-1\right)}\right)\wedge d_{tk}\right\}. \end{array}$$

According to the above definition, the matrix vector strategy execution process is as follows.

1. In this paper, the strategy of clustering matrix is applied to the Apriori algorithm. First, the transaction database *D* is scanned and a clustering matrix *A* is generated for it. If this number of items in this transaction database is *k*, then it is clustered into the matrix *A*(*k*). Each column of the clustering matrix *A*(*k*) represents a different item in the column, and each row represents a detailed convert record containing item sets, and the Boolean quantities 0 and 1 in the matrix indicate whether the item has a record in the matrix or not, respectively, with a record of 1 and no record of 0. The column vectors in the matrix are calculated using the logical operation “AND,” The support degree of each item is calculated by formula (5). According to the calculation result, the frequent item set 1-itemset *L*_1_ is finally determined.
2. *L*_*k*−1_ (*k* ≥ 2) self-join produces the set of the candidate item set *C*_*k*_.
3. Sum the column vectors of the cluster matrix using the “AND” operation. If the support obtained after the “AND” operation of the cluster matrix meets the set threshold value, the item set is directly put into the set *L*_*k*_ of frequent-item set *k*-item. Otherwise, the corresponding column vector “AND” operation is performed on the cluster matrix *A*(*k*+1), and the result is accumulated with the previous support frequency. When the set min_supp threshold is not greater than the accumulated support, the subsequent clustering matrix continues to be scanned until the accumulated support is greater than the set min_supp threshold, and the subsequent matrix ends scanning.

#### 3.1.2. Pruning Strategy

The Apriori algorithm uses *L*_*k*−1_ self-join to generate a set *C*_*k*_ of candidate item sets. In the course of self-join, a large number of infrequent item sets are inevitably generated, and if the algorithm can determine that some items are infrequent item sets according to some rules before generation of *C*_*k*_, it can cut out this part of item sets in advance, which saves their self-join operation and reduces the time to calculate their support frequency. When scanning the database, the pruning strategy reduces the number of frequent item sets generated and reduces the time complexity of the algorithm execution. The pruning strategy is suitable for frequent item sets with the following properties.

**Property 1 .**

If all subsets contained in *A* set are frequent item sets, then *A* set must be frequent item sets.

**Property 2 .**

Among *k*-itemset *A*={*a*_1_, *a*_2_,…, *a*_*k*_}, if there are items *i* ∈ *A* and |*L*_*k*−1_(*i*)| < *i* − 1, then |*L*_*k*−1_(*i*)| represents the number of items *i* contained in the set *L*_*k*−1_.

Based on the above properties, the pruning strategy implementation process is as follows:

1. Calculate |*L*_*k*−1_(*i*)|
2. Calculate the frequencies of all items and record the items with frequencies less than *k* − 1, noted as *A*={*i*|*L*_*k*−1_(*i*)| < *i* − 1}
3. Delete all frequent item sets containing *A* any of the elements in *L*_*k*−1_ and record as L_*k*−1_′
4. Candidate set *C*_*k*_′ is obtained by self-joining of set *L*_*k*−1_′

During the implementation of the pruning strategy, the pruning strategy with the Apriori algorithm can be used after the self-join *L*_*k*−1_′ to further reduce the number of candidate item sets generated again. The time required for frequent item sets when joined is reduced by the prepruning strategy, and the workload is also reduced for the implementation of postpruning. After implementing the prepruning and postpruning strategies, candidate item sets are reduced. This to some extent reduces the time overhead during the database scanning process when calculating the support.

### 3.2. Algorithm Flow and Examples

#### 3.2.1. Execution Process

The algorithm proposed in this paper adds project constraints, matrix-vector strategy, and pruning strategy to the traditional Apriori algorithm. The specific implementation process is as follows:

  Step 1: by scanning the transaction database *D* , the number of items in *D* is obtained, and the matrix is clustered to obtain the *A* matrix. If the matrix contains *k* items, the clustering matrix *A*(*k*) is obtained.
  Step 2: add and sum the vector values of each column in the matrix, calculate the support frequency of the items, and add the items that meet the minimum support threshold value to *L*_1_ and produce a frequent 1-item set.
  Step 3: perform operations on *L*_*k*−1_ with the help of the prepruning strategy, record the number of occurrences of the obtained items in the itemset, delete all infrequent item sets whose support frequency is less than the item *k* − 1 , and record the obtained set as *L*_*k*−1_′.
  Step 4: a self-connection operation is performed on *L*_*k*−1_′, and the connection conditions can be appropriately added to the set constraint items (hypertension, diabetes, etc.), and a candidate *k*-item set *C*_*k*_′ is generated at this time.
  Step 5: after pruning *C*_*k*_′ with the properties of the traditional Apriori algorithm to generate *C*_*k*_, the irrelevant items are reduced.
  Step 6: the length of each item set in the generated itemset *C*_*k*_ is recorded as *k*, so there is no need to consider the clustering matrix whose length is smaller than *k*.The column vectors in the clustering matrix *A*(*k*) are subjected to “AND” operation to obtain the corresponding column vectors for each candidate item set, and the sum of the column elements in the clustering matrix is counted to calculate the support of the corresponding candidate item set. If the minimum support threshold value is less than the support of the candidate items, the set will be added to *L*_*k*_. If the minimum support threshold value is greater than the support of the candidate items, the column vectors in the *A*(*k*+1) will be processed to find the support frequency of the item set and added to the count until the support is not less than the set minimum support threshold value, or all the items in the cluster matrix are scanned.
  Step 7: repeat execution of step 3 to step 6 until *L*_*k*_ is empty to determine the frequent item set *C*_*k*_

#### 3.2.2. Algorithm Implementation Process

In Table 2, database *D* exists and min_supp  = 2. The generation process of frequent item sets is as follows.

(1) Scan the transaction database and generate three clustering matrices based on the number of items contained, denoted by *A*(1), *A*(2), and *A*(3), respectively, and the matrix for each item expressed as a Boolean value is as follows:
  (8) $$\begin{array}{c} A\left(1\right)=\left|\begin{array}{ccccc} 1 & 0 & 1 & 0 & 0\\ 0 & 1 & 1 & 0 & 0\\ 1 & 0 & 1 & 0 & 0\\ 0 & 1 & 1 & 0 & 0\\ 0 & 1 & 0 & 1 & 0 \end{array}\right|,\\ A\left(2\right)=\left|\begin{array}{ccccc} 1 & 1 & 1 & 0 & 0\\ 1 & 1 & 0 & 1 & 0\\ 1 & 1 & 0 & 0 & 1 \end{array}\right|,\\ A\left(3\right)=\left|\begin{array}{ccccc} 1 & 1 & 1 & 0 & 1 \end{array}\right|. \end{array}$$
The support of the item *a*_1_ is as follows: support_*c*(*a*_1_) = ∑_*n*=1_^5^*d*_2*n*1_ = 2 ≥ 2, where the *d*_*knj*_ denotes the Boolean value of the *k* th row and *j* th column of the matrix *A*_*k*_. Similarly, the support of *a*_2_ and *a*_3_ can be calculated as 3 and 4, and both are greater than the minimum support threshold value. The support of the item *a*_4_ is as follows: support_*c*(*a*_4_) = ∑_*n*=1_^5^*d*_2*n*4_ = 1 ≤ 2, the support of the item a_4_ is less than the minimum support threshold value, so the support of the item *a*_4_ in *A*(1) is calculated, and the result is added to the previous calculation, and the result is as follows: support_*c*(*i*_4_) = ∑_*n*=1_^5^*d*_3*n*4_ + ∑_*n*=1_^5^*d*_2*s*4_ = 2. According to the same method, the support of *a*_5_ can be found as 2. The final 1-item set L_1_ is obtained as follows: {*a*_1_}, {*a*_2_}, {*a*_3_}, {*a*_4_} and {*a*_5_}.
(2) After self-join, C_2_ are as follows: {*a*_1_, *a*_2_}, {*a*_1_, *a*_3_}, {*a*_1_, *a*_4_}, {*a*_1_, *a*_5_}, {*a*_2_, *a*_3_}, {*a*_2_, *a*_4_}, {*a*_2_, *a*_5_}, {*a*_3_, *a*_4_}, {*a*_3_, *a*_5_} and {*a*_4_, *a*_5_},
  (9) $$\begin{array}{c} \mathrm{support}\_c\left(\left\{a_{1},a_{4}\right\}\right)=\sum_{n-1}^{m}\left(d_{2n1}\wedge d_{2n4}\right)+\sum_{n-1}^{m}\left(d_{3n1}\wedge d_{3n4}\right)+\sum_{n-1}^{m}\left(d_{4n1}\wedge d_{4n4}\right)=0+1+0=1\leq 2,\\ \mathrm{support}\_c\left(\left\{a_{3},a_{4}\right\}\right)=\sum_{n-1}^{m}\left(d_{2n3}\wedge d_{2n4}\right)+\sum_{n-1}^{m}\left(d_{3n3}\wedge d_{3n4}\right)+\sum_{n-1}^{m}\left(d_{4n3}\wedge d_{4n4}\right)=0+0+0=0\leq 2,\\ \mathrm{support}\_c\left(\left\{a_{4},a_{5}\right\}\right)=\sum_{n-1}^{m}\left(d_{2n4}\wedge d_{2n5}\right)+\sum_{n-1}^{m}\left(d_{3n4}\wedge d_{3n5}\right)+\sum_{n-1}^{m}\left(d_{4n4}\wedge d_{4n5}\right)=0+1+0=1\leq 2,\\ \mathrm{support}\_c\left(\left\{a_{3},a_{5}\right\}\right)=\sum_{n-1}^{m}\left(d_{2n3}\wedge d_{2n5}\right)+\sum_{n-1}^{m}\left(d_{3n3}\wedge d_{3n5}\right)+\sum_{n-1}^{m}\left(d_{4n3}\wedge d_{4n5}\right)=0+1+0=1\leq 2. \end{array}$$
And you can see that in the calculation, {*a*_3_, *a*_5_} and {*a*_4_, *a*_5_} are not satisfied with the set threshold value. The support of the candidate item sets {*a*_1_, *a*_2_}, {*a*_1_, *a*_3_}, {*a*_2_, *a*_3_}, {*a*_2_, *a*_4_}, {*a*_2_, *a*_5_} and {*a*_1_, *a*_5_} are both greater than 2, satisfying the set condition. Thus, the generated frequent 2-item set *L*_2_ is obtained as follows: {*a*_1_, *a*_2_}, {*a*_1_, *a*_3_}, {*a*_2_, *a*_3_}, {*a*_2_, *a*_4_}, {*a*_1_, *a*_5_} and {*a*_2_, *a*_5_}.
(3) Use the prepruning strategy, the number of each item in *L*_2_ is calculated as as follows: |*L*_2_(*a*_1_)|  = 3, |*L*_2_(*a*_2_)|  = 4, |*L*_2_(*a*_3_)|  = 2, |*L*_2_(*a*_4_)|  = 1and |*L*_2_(*a*_5_)|  = 3. In the frequent 2-item set, the occurrences number of a_4_ is not greater than 2, so a_4_ will be deleted and *L*_2_′ are obtained as follows: {*a*_1_, *a*_2_}, {*a*_1_, *a*_3_}, {*a*_1_, *a*_5_}, {*a*_2_, *a*_3_} and {*a*_2_, *a*_5_}. Perform self-join for *L*_2_′, the candidate item set *C*_3_′ are obtained as follows: {*a*_1_, *a*_2_, *a*_3_}, {*a*_1_, *a*_2_, *a*_5_}, {*a*_1_, *a*_3_, *a*_5_} and {*a*_2_, *a*_3_, *a*_5_}; if the prepruning strategy is not used, the candidate 3-item set is obtained as follows: {*a*_1_, *a*_2_, *a*_3_}, {*a*_1_, *a*_2_, *a*_5_}, {*a*_1_, *a*_3_, *a*_5_}, {*a*_1_, *a*_3_, *a*_4_}, {*a*_2_, *a*_3_, *a*_5_} and {*a*_2_, *a*_4_, *a*_5_}. According to the above calculation, 6 candidate item sets are generated before using the former pruning strategy, and 4 candidate 3-item sets are obtained after using the former pruning strategy. In a database with only 9 items, 2 candidate item sets are reduced by using the one-time pruning strategy. When the transaction database is larger, the performance of using the pruning strategy is more obvious strategy. Perform postpruning for the candidate 3-item set, then the candidate item set *C*_3_′ is obtained as follows: {*a*_1_, *a*_2_, *a*_3_} and {*a*_1_, *a*_2_, *a*_5_}.
(4) Calculate the support of the candidate item set *C*_3_ because the number of transactions of the candidate item set is 3, so the frequent item set only needs to be calculated from the clustering matrix *A*(3). Because the support of {*a*_1_, *a*_2_, *a*_3_} is 2 and the support of {*a*_1_, *a*_2_, *a*_5_} is 2, both satisfy the set minimum support threshold value, so *L*_3_ is as follows: {*a*_1_, *a*_2_, *a*_3_} and {*a*_1_, *a*_2_, *a*_5_}.
(5) Perform prepruning strategy for *L*_3_, *L*_3_ is empty and the algorithm ends. The set of all frequent item sets is as follows: {*a*_1_, *a*_2_, *a*_3_} and {*a*_1_, *a*_2_, *a*_5_}.

It can be seen from the above example of algorithm execution that when the traditional Apriori algorithm generates a frequent item set L_3_, it needs to scan the transaction database three times, and the algorithm, after the pruning strategy, only scans the database once. From the perspective of time consumption, it takes less time, and from the perspective of data mining efficiency, the efficiency is improved.

## 4. Experiments

From the content of the previous section, it can be seen that the algorithm has good advancements, and the advantages of the algorithm will be verified below. The environment of this experiment uses a Pentium(R) 2.40 GHz/3.0 GB microcomputer (operating system is Win 7), the simulation environment uses MATLABR2012a, and the data set of the experiment uses Mushroom of the UCI standard test data set, which contains 8, 124 records, each record has 23 attributes, and each attribute has 12 enumeration values.

1. The experiments of setting the two algorithms are carried out under the premise of the same data set and different support thresholds, and the number of generated candidate item sets is shown in Figure 2.
2. Observing Figure 2, we can see that when the min_sup*p* threshold increases from 10 to 30, the number of candidate item sets for the optimization algorithm is reduced from 670 to 256, and the number of candidate item sets for the traditional Apriori algorithm is reduced from 820 to 385. The number of sets is decreasing. However, under the same min_sup*p*, the number generated by the optimization algorithm is significantly lower than that of the traditional Apriori algorithm. Therefore, the optimization algorithm has obvious advantages.
3. The experiment of setting the two algorithms is carried out under the premise of the same data set and different support thresholds. The execution time of the two algorithms is shown in Figure 3.
4. Observing Figure 3, we can see that the min_sup*p* threshold increased from 10 to 40, the execution time of the optimized algorithm decreased from 112 to 40, and the execution time of the traditional algorithm decreased from 175 to 75. The execution time of both algorithms is decreasing. However, under the same min_sup*p*, the execution time of the optimization algorithm is significantly lower than that of the traditional Apriori algorithm, so the optimization algorithm has obvious advantages.
5. Under the premise of min_sup*p*  = 0.3 and different numbers of datasets, the execution time of the two algorithms is shown in Figure 4.

Observing Figure 4, we can see that the number of datasets increased from 2000 to 8000, the execution time of the optimized algorithm increased from 25 to 55, the execution time of the traditional algorithm increased from 32 to 81, and the execution time of both algorithms increased. However, under the same dataset, the execution time of the optimization algorithm is significantly lower than that of the traditional Apriori algorithm, so the optimization algorithm has obvious advantages.

## 5. Conclusions

This paper proposes a project under the constraint condition of clustering matrix and the pruning strategy of combining the association rule data mining algorithm, the algorithm is applied in setting project constraints under the premise of clustering matrix and the method of pruning strategy largely reduced the number of algorithms to generate candidate item sets, avoid the I/O overhead of the problems of multiple scanning database, and improve the execution efficiency of the algorithm. The simulation experiment is verified from three aspects. It can be seen from the experimental results that the number of candidate sets generated by the optimized Apriori algorithm under different support threshold conditions is less than that of the traditional algorithm, and the execution time of the algorithm is greatly reduced, thereby improving the execution efficiency of the algorithm. At present, the association rules generated by the algorithm in this paper are given in a formal formula, which is inconvenient for users to understand. In future work, the visualization of the data mining process will be studied.

## Figures and Tables

**Figure 1:** Add a mining for user constraints.

**Figure 2:** Candidate sets for different support threshold generation.

**Figure 3:** Candidate item sets at different support thresholds.

**Figure 4:** Execution time under different number of data sets.

**Table 1:** Define symbols.

*k*-item	The set of *k* items

*L*_*k*_	min_supp item Sets
*C*_*k*_	Candidate item sets

**Table 2:** Database.D

Item	Item sets
*A*1	*a*_1_, *a*_2_, *a*_5_
*A*2	*a*_2_, *a*_4_
*A*3	*a*_2_, *a*_3_
*A*4	*a*_1_, *a*_2_, *a*_4_
*A*5	*a*_1_, *a*_3_
*A*6	*a*_2_, *a*_3_
*A*7	a_1_, *a*_3_
*A*8	a_1_, *a*_2_, *a*_3_, *a*_5_
*A*9	a_1_, *a*_2_, *a*_3_

## Data Availability

The data used in the experiment are obtained from the UCI standard test dataset of the Mushroom data.
